The article "Synthesis and Workability Behavior of Cu-X wt.% TiC (x = 0, 4, 8, and 12) Powder Metallurgy Composites" was retracted in 2023. Reasons: signs of a paper mill; suspected computer-generated content; unreliable results or conclusions; concerns about the data.

# Synthesis and Workability Behavior of Cu-X wt.% TiC (*x* = 0, 4, 8, and 12) Powder Metallurgy Composites

**DOI:** 10.1155/2022/8101680

**Published:** 2022-05-21

**Authors:** V. Mohanavel, M. Ravichandran, K. S. Ashraff Ali, T. Sathish, Alagar Karthick, S. Arungalai Vendan, Palanivel Velmurugan, Saleh H. Salmen, Saleh Alfarraj, S. Sivakumar, Atkilt Mulu Gebrekidan

**Affiliations:** ^1^Centre for Materials Engineering and Regenerative Medicine, Bharath Institute of Higher Education and Research, Chennai, 600073 Tamil Nadu, India; ^2^Department of Mechanical Engineering, Chandigarh University, Mohali 140413, Punjab, India; ^3^Department of Mechanical Engineering, K. Ramakrishnan College of Engineering, Trichy-621112, Tamil Nadu, India; ^4^Department of Mechanical Engineering and University Centre for Research & Development, Chandigarh University, Mohali 140413, Punjab, India; ^5^Department of Mechanical Engineering, C. Abdul Hakeem College of Engineering and Technology, Vellore 632509, Tamil Nadu, India; ^6^Department of Mechanical Engineering, Saveetha School of Engineering, SIMATS, Chennai 602 105, Tamil Nadu, India; ^7^Department of Electrical and Electronics Engineering, KPR Institute of Engineering and Technology, Coimbatore 641407, Tamil Nadu, India; ^8^Department of Electronics and Communication, Dayananda Sagar University, Bengaluru, Karnataka, India; ^9^Department of Botany and Microbiology, College of Science, King Saud University, PO. Box 2455, Riyadh 11451, Saudi Arabia; ^10^Zoology Department, College of Science, King Saud University, Riyadh 11451, Saudi Arabia; ^11^Department of Bioenvironmental Energy, College of Natural Resources and Life Science, Pusan National University, Miryang-si 50463, Republic of Korea; ^12^Department of Mechanical Engineering, Faculty of Mechanical Engineering, Arba Minch Institute of Technology (AMIT), Arba Minch University, Arba Minch, Ethiopia

## Abstract

In this work, copper (Cu) matrix composite reinforced with titanium carbide (TiC) was fabricated by powder metallurgy (PM) method with the varying TiC content from 0% to 12% by weight in the step of 4%. The required weight percentage of powders was milled in an indigenously developed ball milling setup. Green compacts were made using a computer-controlled hydraulic press (400 kN) and sintered in a muffle furnace at a temperature of 950°C. Scanning electron microscope (SEM) was used to analyze the distribution of TiC particles in Cu matrix in as-sintered conditions. X-ray diffraction (XRD) analysis resulted in the existence of respective phases in the produced composites. The structural characteristics such as stress, strain, dislocation density, and grain size of the milled composites were evaluated. Cold upsetting was conducted for the sintered composites at room temperature to evaluate the axial (*σ*_*z*_), hoop (*σ*_*ө*_), hydrostatic (*σ*_*m*_), and effective (*σ*_*eff*_) true stresses. These stresses were analyzed against true axial strain (*ε*_*z*_). Results showed that the increase in the inclusion of weight percentage of TiC into the Cu matrix increases density, hardness, (*σ*_*z*_), (*σ*_*ө*_), (*σ*_*m*_), (*σ*_*eff*_), and stress ratio parameters such as (*σ*_*z*_/*σ*_*eff*_), (*σ*_*θ*_/*σ*_*eff*_), (*σ*_*m*_/*σ*_*eff*_), and (*σ*_*z*_/*σ*_*θ*_) of the composites.

The article "Synthesis and Workability Behavior of Cu-X wt.% TiC (x = 0, 4, 8, and 12) Powder Metallurgy Composites" was retracted in 2023. Reasons: signs of a paper mill; suspected computer-generated content; unreliable results or conclusions; concerns about the data.

## 1. Introduction

PM is the one that leads to a paradigm shift in the field of manufacturing. The importance of the PM process was reconnoitered during the nineteenth century during the usage of tungsten powders. Applications of powder metallurgy are not been limited in a particular due to its distinct features in addition to its efficiency, environment-friendly, and economic [1]. Later the industrial needs initiate the researchers toward the processing of different materials through powder metallurgy. Even now, the industrial need in regard to newer materials with tailored properties is not yet resolved and this may be attributed to the help of composite materials. Several modes of the manufacturing process are there, and powder metallurgy is the unique processing technique that helps to synthesize the materials with improved properties. Copper is one of the materials, which has a wide range of usage in powder metallurgy due to its properties like ductility, malleability, and corrosion resistance, electrical, and thermal conductivity [2]. Ceramic particles reinforced copper-based composites are very attractive in recent years due to their wonderful properties such as thermal, electrical, and mechanical properties [3]. Copper composites are widely used in aerospace and automotive drive shafts, ground vehicle brake rotors, and explosive engine components. TiC is one of the important ceramic materials, and it is used in many applications because of its excellent modulus and hardness. TiC is used as reinforcement materials to fabricate the copper-based composite due to its potential applications in many areas [4].

Copper composites up to 5 wt. % of titanium were mixed and sintered and identified that it is possible to make sinters with a theoretical density of 95% [5]. Tribological and mechanical behavior of copper is improved with the nanoalumina by Chen et al. who observed the modifications in microstructure due to the variation in the sintering temperature and arrived at an optimized temperature to achieve better bonding strength [6]. Zhao et al. synthesized the copper composites with iron wire as reinforcement to attain 10 and 17 volume percentages of iron wire and found higher strength and conductivity for 10 volume percentage [7].

The article "Synthesis and Workability Behavior of Cu-X wt.% TiC (x = 0, 4, 8, and 12) Powder Metallurgy Composites" was retracted in 2023. Reasons: signs of a paper mill; suspected computer-generated content; unreliable results or conclusions; concerns about the data.

Hybrid composites with copper, graphite, and silicon carbide were synthesized by Zhan and Zhang to investigate the tribological properties and the improved wear resistance was observed due to the combined effect of reinforcements [8]. Copper composites with silicon carbide particles were synthesized by Shabani et al. and the improved hardness and relative density were found with the sinter-forging method [9]. Copper composites with the alumina reinforced by the niobium particle were synthesized by Srivatsan and Troxell to investigate its strength through tensile testing [10]. Wang et al. synthesized Mg_2_B_2_O_5_ and silicon carbide whiskers reinforced Al composites and observed that the strain rate significantly influences the stress of the composite [11]. Liu et al. synthesized the ZA27 hybrid composites reinforced with whiskers carbon nanotube and aluminum and constructed a dynamic model [12]. Bensam Raj et al. synthesized the aluminum composites reinforced with silicon carbide and examined the outcome of SiC addition on the workability of the produced composite [13].

Fe-C-Mn composites were synthesized through PM by Selvakumar et al. and the higher workability was observed at the initial loading, and furthermore, it tends to be decreased [14]. Copper composites with 7.5% of titanium carbide in two aspect ratios were synthesized by Narayanasamy et al. and found the increased plastic range at the first stage due to the incorporation of TiC [15]. Hybrid copper composites reinforced with titanium dioxide and graphite were synthesized by Ilayaraja et al. and presented the results that the inclusion of reinforcements in matrix enhanced the hardness and strength coefficient of the composites [2]. Ravichandran and Anandakrishnan synthesized hybrid aluminum composites with molybdenum trioxide and optimized the PM parameters to achieve high strength coefficient [16]. Anandakrishnan et al. synthesized the in situ aluminum composites with titanium carbide and studied its forming behavior [17].

Researchers studied the graphite reinforced copper composites and reported that the addition of graphite content after milling improved the wear resistance of the composite samples [18, 19]. Fanyan Chen et al. developed copper composites with graphene as reinforcement materials, and they reported that the inclusion of graphene leads to improvement in mechanical, thermal, electrical, and tribological properties [20]. Yu Bian et al. reported the tribology and microstructure if the Cu/niobium carbide composite developed via PM technique and they observed the improved properties for the composite samples [21]. Manish Dixit and Rajeev Srivastava developed Cu/Gr composite via PM, and they concluded that the even spreading and decent interfacial adhesion increases the physical properties of the composites [22]. Enze Xu et al. used PM approach to produce Cu/Gr composite and obtained outstanding physical and mechanical properties for the composite samples [23].

The article "Synthesis and Workability Behavior of Cu-X wt.% TiC (x = 0, 4, 8, and 12) Powder Metallurgy Composites" was retracted in 2023. Reasons: signs of a paper mill; suspected computer-generated content; unreliable results or conclusions; concerns about the data.

From the above, so far the study of workability behavior of Cu-TiC PM composites is not attempted. Hence, the present work aims to synthesis Cu-TiC composites via the PM method and studies the workability behavior during cold upsetting. The structural properties, density, and hardness of the TiC reinforced copper composites were reported. The objective of this work is to improve the properties and workability of the TiC-reinforced Cu-based composites.

## 2. Experimental Details

Copper powders, 99.0% pure, and TiC powders, 99.95% pure (Kemphasol; Mumbai, India), were selected as matrix and reinforcement materials, respectively. Cu and TiC were weighed inaccurately and then mixed in a ball mill for 5 h. The 10 : 1, ball to powder ratio on a weight basis, was employed. The speed of the drum was 300 rpm. After trial experiments, it was decided to use 300 rpm for the milling operation. Four different kinds of samples were produced: 1) Cu-0 wt.% TiC, 2) Cu-4 wt.% TiC, 3) Cu-8 wt.% TiC, and 4) Cu-12 wt.% TiC. The reason for selecting these compositions is that to analyze the effect of wt. % TiC on the workability behavior of Cu-based composites. Beyond 12 wt. of TiC, the samples were too brittle with high porosity. The milled powders were compacted in a hydraulic press at a pressure of 700 MPa. Zinc stearate was applied to the die wall as a lubricant. The samples were sintered at a temperature of 950°C (2 h) in the furnace, which is Argon-controlled. SEM (JEOL JSM-35 CF SEM) was used to study the microstructure of the prepared samples. PANalytical X'Pert X-ray diffractometer C_u_K*α* target (*λ* = 1.5418 Å) was used to analyze the different phases of the composites. The structural parameters of the sintered composites were determined from the XRD pattern as reported elsewhere [24, 25].

Archimedes method was used to find the density of the sintered and green samples. Brinell hardness was measured using a Brinell hardness machine under an applied force of 1000 N with a 10 mm diameter ball indenter. An average of 5 measurements was taken to measure the hardness of the sintered samples. The upsetting test was conducted at room temperature, and the applied load was increased at the level of 20 kN. The cold upset test setup is shown in Figure 1. The changes in the dimension of the samples were noted. The test was conducted until a fine crack was observed in the samples. The measured dimensions are used to determine the (*σ*_*z*_) (*σ*_*ө*_), (*σ*_*m*_), *(ε*_*z*_), and Poisons ratio (*α*) as reported elsewhere [26]. Cold upset was done to decrease the porosity of the developed composites.

The article "Synthesis and Workability Behavior of Cu-X wt.% TiC (x = 0, 4, 8, and 12) Powder Metallurgy Composites" was retracted in 2023. Reasons: signs of a paper mill; suspected computer-generated content; unreliable results or conclusions; concerns about the data.

## 3. Results and Discussion

### 3.1. SEM Analysis of Sintered C-TiC PM Composite Preforms

Figures 2(a)–2(d) show the SEM images of Cu-TiC sintered PM composite produced via the PM route. Two different regions are observed from the microstructures, and it differentiates the matrix and reinforcement phase. The good homogeneous distribution of reinforcements was obtained by using an indigenously fabricated ball milling setup (Figure 1(a)). Figures 2(a)–2(c) display the even dispersal of 4, 8, and 12 wt. % of TiC in Cu matrix. It is observed from the images that the distance between TiC particles is diminished consistently as the wt. % of TiC particles increased. The size of the reinforcement domain is increased when the percentage of TiC increased. The interface between the Cu matrix and TiC dispersal is undoubtedly detected from the magnified views as shown in Figure 2(d).

### 3.2. XRD analysis sintered Cu-TiC PM composite preforms

The crystal structure of the as-sintered Cu-TiC composites was analyzed by XRD, and the patterns are illustrated in Figure 3. The XRD patterns of Figure 3 exhibit Cu peaks and TiC peaks. The Cu is observed in (111), (200), (220), (311), (222), and (400) planes, and the TiC is observed in (111), (200), and (311) planes. XRD pattern confirms the absence of other intermetallic. The intensity in peak ensures the increase in TiC content in the matrix. The peak broadening is noted in the pattern since the TiC content is increased in wt. basis.

The dislocation density, lattice parameter, crystallite size, lattice macrostrain, and the unit cell volume of Cu-TiC sintered PM composites are provided in Table 1. The grain size is decreased due to the addition of TiC in the copper matrix. The reason is that the initial particle size of the TiC is lower than the Cu particle.  Figure 4 reveals the effect of TiC on the grain size of Cu matrix composites.  Figure 5 reveals the effect of TiC on dislocation density and unit cell volume of Cu matrix composites. The size decreases from 147 nm to 126 nm. However, the lattice strain increased as a function of the particle content. The reason for this could be severe plastic deformation and work hardening of powders by the ball milling process.  Figure 6 reveals the effect of TiC on lattice space and lattice constant of Cu matrix composites.  Figure 7 reveals the effect of TiC on stress and strain of Cu matrix composites. Hence, the increase in dislocation value is evident in the addition of TiC particle in the Cu matrix [27].

The article "Synthesis and Workability Behavior of Cu-X wt.% TiC (x = 0, 4, 8, and 12) Powder Metallurgy Composites" was retracted in 2023. Reasons: signs of a paper mill; suspected computer-generated content; unreliable results or conclusions; concerns about the data.

### 3.3. Effect of TiC on Density of Sintered Cu-TiC PM Composite Preforms

Figure 8 displays the effect of TiC addition on the density of the Cu matrix composites reinforced with 0, 4, 8, and 12 wt. % TiC in as-sintered and cold upset conditions. The density of the composites decreases for the increase in TiC particles. The cause for the decrease in density is due to the unembellished deformation of the particles during the milling stage. The maximum density of the composites has been achieved for 4 wt. % TiC composite. The addition of hard TiC particles resists the densification during compaction, and thus, the decrease in density is observed for Cu-12 wt. %TiC composite. The presence of titanium in the copper matrix produces a solid solution. This makes the milled powder becomes stronger. When compared with the sintered samples, an increase in density was observed for the cold upset sample. The reason could be the complete consolidation and closing of pores during cold upsetting. The decrease in porosity also increases the density of the samples.

### 3.4. Effect of TiC on Hardness of Sintered Cu-TiC PM Composite Preforms

Figure 9 displays the result of the accumulation of TiC particles in the Cu matrix on the hardness of the sintered and cold upset composites. The improvement in hardness is observed for the composite samples due to the incorporation of TiC with an increase in wt.% for both sintered and cold upset samples. The maximum hardness was observed for the Cu-12 wt.% TiC composite, and when compared with Cu-4 wt.% TiC composite, 56% of hardness improvement was obtained. As reported in Table 1, the increase in dislocation density decreases in grain size and work hardening of powders during milling is responsible for the increase in hardness of the composites. When compared with sintered composites, the cold upset composite samples have more hardness.

### 3.5. Workability Behavior of Sintered Cu-TiC PM Composite Performs during Cold Upsetting

Figure 10 has been plotted between the *σ*_*z*_ and *ε*_*z*_ for Cu matrix composite containing TiC particles, namely, 4%, 8%, and 12%. From Figure 4, it is observed that with increasing TiC content, the *σ*_*z*_ increases for any given *ε*_*z*_ value. The increase in *σ*_*z*_ is due to the accumulation of TiC because of more work hardening of Cu matrix. Another cause is that as the TiC increases, the density also rises and the decrease in porosity is observed. Thus, the load transfer capacity is improved due to the TiC accumulation in the copper matrix.

The article "Synthesis and Workability Behavior of Cu-X wt.% TiC (x = 0, 4, 8, and 12) Powder Metallurgy Composites" was retracted in 2023. Reasons: signs of a paper mill; suspected computer-generated content; unreliable results or conclusions; concerns about the data.

The plot is drawn between the *σ*_*θ*_ and the *ε*_*z*_ is exposed in Figure 11. The *σ*_*θ*_ also increases for the rise in TiC content. Cu with 12% TiC content exhibits the highest *σ*_*θ*_, and Cu with 4% TiC displays the lowest *σ*_*θ*_ of all the composites tested. The various stresses have been studied for this composition. The *σ*_*θ*_ was observed for the lowest fracture strain when compared with other stresses.

The plot is drawn among the *σ*_*m*_, the *ε*_*z*_ is revealed in Figure 12, and the same behavior has been observed for all the samples. The maximum *σ*_*m*_ was observed for the composite with high reinforcement content. This stress is due to the true axial and true hoop stress. When the two other stresses increase, the *σ*_*m*_ also increased. The plot is drawn between the *σ*_*eff*_, the *ε*_*z*_ is revealed in Figure 13, and the same behavior has been observed. *σ*_*eff*_ is a significant feature that extremely affects the workability constraint, established during deformations.

### 3.6. Strength Coefficient versus Strain Hardening Index

Figure 14 displays the outcome of the accumulation of TiC on the strength coefficient (K) and strain hardening index (n). The “K” and “n” values are found from the curve fitting obtained for *σ*_z_ versus *ε*_z_. The “K” increases for the increase in addition of TiC and the “n” decreases. The reasons are that the accumulation of hard TiC particles rises the dislocation density and the resistance of the deformation is improved, and thus, the strength of the composites is increased for the rise in incorporation of TiC particles in the Cu matrix. The decrease in “n” is obtained for the composite with TiC. The hard reinforcement particles fight against deformation during loading (Figure 2(a)).

### 3.7. Analysis of Stress Ratio Parameters

Figures 15–17 had been drawn among the (*σ*_*z*_/*σ*_*eff*_), (*σ*_*θ*_/*σ*_*eff*_), and the *ε*_*z*_ for sintered Cu-TiC composites during cold upsetting.  Figure 15 displays the plot among (*σ*_*z*_/*σ*_*eff*_) and *ε*_*z*_. This figure shows the rise in stress ratio parameter (*σ*_*z*_/*σ*_*eff*_) with an increase in TiC particles in the Cu-TiC composite. Among the various composites tested, the higher stress ratio parameter (*σ*_z_/*σ*_eff_) was observed for Cu-12 wt.% TiC composite. The addition of hard particles increases the dislocation density (Table 1) and resists the deformation during cold upsetting; thus, the induced stress also increased. In the present study, the stress ratio parameter decreases for the increase in the true axial strain. The reason is that the rate of increase in true effective stress (*σ*_eff_) is higher than that of increase in true axial strain (*ε*_*z*_). Figures 16 and 17 show the relationship between the (*σ*_*θ*_/*σ*_eff_), (*σ*_*m*_/*σ*_eff_), and the (*ε*_*z*_). From Figures 16 and 17, it is observed that the trend is similar to that is observed in Figure 15. It means that all the stress ratio parameters rise with the rise in the addition of TiC particles in the composites during cold upsetting. The increase in strength coefficient also increases the stress ratio parameter.

The article "Synthesis and Workability Behavior of Cu-X wt.% TiC (x = 0, 4, 8, and 12) Powder Metallurgy Composites" was retracted in 2023. Reasons: signs of a paper mill; suspected computer-generated content; unreliable results or conclusions; concerns about the data.

Figure 18 displays the graph among (*σ*_*θ*_/*σ*_*m*_) and (*ε*_*z*_) during cold upsetting of Cu-TiC composites. The increased (*σ*_*θ*_/*σ*_*m*_) is observed for the increase in TiC particles and increase in (*ε*_*z*_). The reason is that the induced true hydrostatic stress (*σ*_*m*_) is less than the induced (*σ*_*θ*_) during plastic deformation for the sintered Cu-TiC composites.

## 4. Conclusions

The following conclusions can be drawn from the present investigations:

- SEM studies of sintered composites exhibited homogeneous microstructure of samples with fine TiC additions and typically distributed at copper particle matrix.
- XRD analysis reveals the occurrence of TiC particles and ensures the no other intermetallic is found during sintering.
- The hardness of the sintered and cold upset composites increases for the TiC reinforced composite samples. When compared with sintered samples, the high hardness was observed for the cold upset composite samples.
- The density of sintered Cu-TiC powder metallurgy composites decreases for the increase in weight percentage of TiC content. The density of cold upset samples is higher than the as-sintered samples.
- The addition of TiC particles in the milled Cu-TiC composites powders decreases the particle size and increases the dislocation density, lattice strain, and unit cell volume.
- The workability of the Cu-TiC composites decreases for the increase in weight percentage of TiC and the increased in true axial stress (*σ*_*z*_), true hoop stress (*σ*_*θ*_), true hydrostatic stress (*σ*_*m*_), and true effective stress (*σ*_eff_) were observed during cold upsetting.

## Figures and Tables

**Figure 1:** (a) Cu-TiC sintered composite preforms. (b) Cu-TiC composite preform during cold upsetting between flat dies.

**Figure 2:** SEM images of (a) Cu-4% TiC, (b) Cu-8% TiC, (c) Cu-12% TiC composites (20 *µ*m scale), and (d) Cu-12% TiC composites (10-*μ*m scale).

**Figure 3:** XRD analysis of (a) Cu-0% TiC, (b) Cu-4% TiC, (c) Cu-8% TiC, and (d) Cu-12% TiC sintered PM composites.

**Figure 4:** Effect of TiC on the grain size of Cu matrix composites.

The article "Synthesis and Workability Behavior of Cu-X wt.% TiC (x = 0, 4, 8, and 12) Powder Metallurgy Composites" was retracted in 2023. Reasons: signs of a paper mill; suspected computer-generated content; unreliable results or conclusions; concerns about the data.

**Figure 5:** Effect of TiC on dislocation density and unit cell volume of Cu matrix composites.

**Figure 6:** Effect of TiC on lattice space and lattice constant of Cu matrix composites.

**Figure 7:** Effect of TiC on stress and strain of Cu matrix composites.

**Figure 8:** Effect of TiC on the density of sintered and cold upset Cu matrix composites.

**Figure 9:** Effect of TiC on hardness sintered and cold upset Cu matrix composites.

**Figure 10:** True axial stress (*σ*_*z*_) versus true axial strain (*ε*_*z*_).

**Figure 11:** True hoop stress (*σ*_*θ*_) versus true axial strain (*ε*_z_).

**Figure 12:** True hydrostatic stress (*σ*_m_) versus true axial strain (*ε*_z_).

**Figure 13:** True effective stress (*σ*_eff_) versus true axial strain (*ε*_z_).

**Figure 14:** Effect of TiC addition on strength coefficient and strain hardening index.

**Figure 15:** Stress ratio parameter (*σ*_*z*_/*σ*_eff_) versus true axial strain (*ε*_*z*_).

**Figure 16:** Stress ratio parameter (*σ*_*θ*_/*σ*_eff_) versus true axial strain (*ε*_*z*_).

**Figure 17:** Stress ratio parameter (*σ*_m_/*σ*_eff_) versus true axial strain (*ε*_*z*_).

**Figure 18:** Stress ratio parameter (*σ*_*z*_/*σ*_*θ*_) versus true axial strain (*ε*_*z*_).

**Table 1:** Structural characteristic of (a) Cu-0% TiC, (b) Cu-4% TiC, (c) Cu-8% TiC, and (d) Cu-12% TiC sintered PM composites.

Sl. no.	Lattice spaced Å	Lattice constant (a) Å	Grain size (s) nm	Strain (*ε*) X10^−3^	Stress 10^10^	Dislocation density (*ρ*_*D*_) X10^14^, m^2^	Unit cell volume (V), Å^3^
1	1.4894	3.5371	156.87	0.4761	0.1724	4.257	71.214
2	1.5484	3.6637	147.95	0.4175	0.1906	4.4119	79.3885
3	1.5953	3.8111	143.30	0.4099	1.8567	4.6811	88.6436
4	1.6034	3.9294	136.611	0.3852	4.2528	6.4422	96.8598

## Data Availability

The data used to support the findings of this study are included in the article and available from the corresponding author upon request.
